# Effects of Occupational Therapy Program Based on Active Meditation on Hair Cortisol Levels in Undergraduate Healthcare Students

**DOI:** 10.1155/2022/2174397

**Published:** 2022-06-08

**Authors:** Alejandra Espinosa, Rodolfo Morrison, Diego Gonzalez, Juan Jamardo, Federico Fortuna, Carmen-Paz Díaz, Pamela Gutiérrez, Carla Frías, Paula Soto, Alejandra González, Sandra Mella, Bibiana Fabre

**Affiliations:** ^1^Escuela de Medicina, Campus San Felipe, Universidad de Valparaíso, Chile; ^2^Universidad de Chile, Facultad de Medicina, Departamento de Tecnología Médica, Santiago, Chile; ^3^Universidad de Chile, Facultad de Medicina, Departamento de Terapia Ocupacional y Ciencia de la Ocupación, Santiago, Chile; ^4^Universidad de Buenos Aires, Facultad de Farmacia y Bioquímica, Departamento de Bioquímica Clínica, Cátedra de Bioquímica Clínica I, Buenos Aires, Argentina; ^5^Universidad de Chile, Facultad de Ciencias Sociales, Carrera de Trabajo Social, Santiago, Chile; ^6^Universidad del Desarrollo, Facultad de Medicina-Clínica Alemana, Carrera de Terapia Ocupacional, Santiago, Chile

## Abstract

**Methods:**

Undergraduate students from the University of Chile's health careers were divided at random into control (*n* = 7) and treated groups (*n* = 15). The treated group participated in an active meditation program once a week for three months. This treatment included different techniques such as Chakra Sounds, Nataraj, Mandala, Kundalini, Devavani, Gourishankar, and Nadabrahma. Hair samples were taken before and after the treatment period to measure cortisol.

**Results:**

The control group increased cortisol level 168.9 ± 76.8 pg/mg compared with initial levels. The treated group shows a decrease of initial cortisol values in 28.5 ± 12.8 pg/mg after meditation protocol application.

**Conclusions:**

Blending active meditation in students' daily routine through occupational therapy intervention might prevent undergraduate students' stress in healthcare careers.

## 1. Introduction

A recent study performed on undergraduate students from Chile's medical careers shows that 98% of them present stress signs [1]. This social disease is an important reason to evaluate meditation practices in the students' daily routine to contribute to better social and physical environments capable of decreasing anxiety and stress [2, 3]. Meditation is considered a powerful tool against stressful situations; several studies have demonstrated a significant quality of life improvement in different populations [4]. Anxiety decrease, cognitive performance increase, and beneficial physiological brain changes are described among its benefits [5, 6]. Mindfulness practices, which incorporate a meditation as a center, reduce high blood pressure in hypertensive subjects and stress levels in patients with cardiovascular diseases [7]. Besides, neck and back chronic pain and headache by tension decrease with meditation practice [8, 9]. Najafidoulatabad et al. have shown that yoga training program for mind control through meditation improves physical performance, satisfaction, and sexual function in women with multiple sclerosis [10]. Moreover, people who continuously practice meditation have a low rate of mental disorders such as depression, stress, and anxiety [11]. Vadiraja et al. showed that the addition of a meditation inside of a yoga program significantly decreases anxiety, depression, and stress [12]. Furthermore, morning cortisol levels decreased in the meditation and yoga-treated group compared with controls in a breast cancer population. In young people, meditation also induces general well-being by treating various symptoms present in psychiatric disorders, improving mental and physical health [13, 14]. Meditation gives several benefits under 18-year-old people, favoring conflict resolution and stress well-management [15, 16] and emotional control [17]. School-based mindfulness has shown a reduced risk of developing suicidal ideation and self-harming and showed an improvement in attentional self-regulation in the treatment of neurodevelopmental disorders such as attention-deficit disorder [18].

Meditation is based on taking notice to each experience set in the body at the present moment. It is characterized by being aware of any part and function of the body. The practice of meditation often develops this capacity. In addition, meditation training improves attention and self-regulation systems, providing different skills in individuals with attention disorders. Meditative practices have been extensively studied in recent decades, including meta-analyses concluding that the main benefit is the improvement of executive function and emotion dysregulation, present in attention deficit hyperactivity disorder [17–19].

Meditation practice includes different schools and techniques. The most common is passive meditation, which generally involves being still and sitting in a comfortable place with the back straight. As an induction, brief verbal commands are usually given, such as paying attention to the breath and letting thoughts pass without getting involved [20].

In the current research, active meditation effect was studied, incorporating the active movement of the whole body [21]. Active meditation, particularly the proposed one by Osho, includes various physical movements such as dance, or simply “letting oneself be carried away” by different sounds. It focuses on making the body experience movements that it does not perform daily. Some examples can be running without moving on the same point, singing melodies in a group, breathing and holding the air as much as possible, performing hand movements in sync with an instructor, and among many other steps. Most of these techniques are integrated into subtypes of active meditation and have three or four stages [22].

The meditation techniques used in this research were:

- *Nadabrahma Meditation*. This is done by sitting down and consists of four steps. The first one consists of the simulation of insect buzzing sound through the mouth; in the second one, a slow pattern is followed with the hands led by the guide; and in the third one, silence is maintained
- *Gourishankar Meditation*. This kind of meditation has four steps. Sitting with eyes closed is required in the first one, and then, deep inhalation through the mouth, followed by a held breath as long as possible, is necessary. Then, exhale slowly through the mouth and leave the lungs as empty as possible. The following step, breathing with a normal rhythm, the fire of a burning candle is observed. Subsequently, the “Latiham” is performed, which corresponds to standing up and letting oneself be carried away by the movements that the body itself wants to perform. Finally, the person is lying down with eyes closed, and silence is maintained
- *Kundalini Meditation*. In this meditation, which has four stages, the body must be shaken energetically. Afterward, a dance phase begins. Subsequently, it remains motionless, standing or sitting. Finally, the person is lying down, keeping closed eyes, without movement
- *Nataraj Meditation*. People must dance keeping closed eyes and letting themselves be carried away by the music. Then, it is necessary to lie down with eyes closed and remain motionless and silent. Afterward, the dance turns once again
- *Mandala Meditation*. With eyes open, begin to run in one place, without moving forward, raising knees as high as possible. Then, sitting down and with eyes closed, circular movements are made with the upper part of the body, keeping the support point on sit bones. Then, lying on their backs and with their eyes open, begin to move eyes in circles to the right. Finally, stop and close the eyes in the same position
- *Devavani Meditation*. In this meditation, at first, remain motionless listening to music. Next, sitting down and with eyes closed, they are instructed to make meaningless sounds in a soft tone. Then, continue to make a sound, but it is necessary to stand up and begin the Latiham (described above). To finish, in silence, it is necessary to lie on your back
- *Chakra Sounds*. This meditation consists of making sounds out loud, accentuating the concentration in different parts of the body (where different “chakras” (The chakras are understood as energy centers located in and around the human body. In Eastern philosophy, it is understood that there are 7 main ones, each with its own location and name: the base of the spine is muladhara; the lower abdomen is svadhisthana; the chest is manipura; the heart, anahata; the throat, visuddha; the forehead, ajna; and the crown of the head, sahasrara [23].) would be found). It is by done standing or lying down. End by keeping quiet in a comfortable position

All these techniques have a duration of 1 hour.

Active meditation is an alternative to the traditional physical-passive meditation practices focusing on achieving well-being through body movement. So far, there are very few studies about active meditation effectiveness on controlled trials [21, 24]. We have previously shown some promissory results of this practice on physical and stress-altered psychomotor markers [25]. We aimed to evaluate whether incorporating active meditation practices in the dairy routine could reduce chronic stress in undergraduate students, using the hair cortisol as a biomarker. Hair cortisol concentration is highly correlated with exposure to chronic stressful events [26]. Considering that hair grows on average 1 cm per month, 3 cm of hair has individual cortisol accumulated during the last three months [27].

In order to modify the daily activities, occupational therapy approach using meditation was incorporated as a mandatory activity twice a week, promoting occupational balance [28] where active meditation is included as part of students' routine.

## 2. Material and Methods

### 2.1. Participants

Undergraduate students from the University of Chile's health careers were invited to participate in a three-month active meditation course (18 sessions, 1 hour, and 30 min. each one) by an open called. The sample size was defined based on those who agreed to participate and completed the participation requirements. Twenty-two students agreed to participate in this study. Seven of them constituted the control group, participating in a painting course, so to the experimental group was integrated by 15 students. All 15 students in the intervention group participate in the same sequence of meditation. The control group was already participating in a painting course at the university. They were interested in the subject, but for the 7, it was a new activity.

Treatment and control groups were integrated by males and females (Table 1). None of them have meditation experience. There ages were between 18 and 22 years, and the students were distributed in different years of training (Table 2). We assume that both groups have similar levels of stress (Table 3) and similar life situations, but this was not evaluated with any instrument.

### 2.2. Occupational Therapy Intervention Based on Active Meditation

Meditation practice was incorporated by occupational therapy interventions focusing on routine structuration and time management. In the initial sessions, a qualitative evaluation of each student perception regarding their routine was performed. Later, goals were decided according to how they sought to modify the most problematic aspects in their routine. Guidelines were given for routine management based on the Human Occupation Model. Small discussion groups were held in each session to share progress in the routine reorganization process. The use of active meditation as a tool for managing stressful situations was intended. Four sessions were used to organize the routine structuration. Active meditation sessions were once a week and were included in daily routine, using different techniques (*Nadabrahma*, *Gourishankar*, *Kundalini*, *Nataraj*, *Mandala*, *Devavani*, and *Chakra Sounds).* A reflection period about meditation usefulness in daily routine was incorporated at the end of each meditation session.

### 2.3. Biological Sample

Hair samples were collected previously at the start of the courses and after the 18 active meditation sessions. Hair samples were collected using scissors from the posterior vertex as close to the scalp as possible, taking three cm from each participant to evaluate hair cortisol concentration accumulated during the last three months. Each sample was conserved in aluminum foil at room temperature and then was sent to the endocrinology laboratory, Buenos Aires University, Argentina, for cortisol measurement.

### 2.4. Cortisol Measurement

Each hair sample was considered, and then, cortisol was extracted and measured by an automated chemiluminescent method (Immulite 2000 autoanalyzer, Siemens, LA, USA) according to the standardized protocol reported by Gonzalez et al. The cortisol concentration was expressed in pg/mg hair. Hair cortisol concentration reference interval in healthy individuals with low levels of stress was 40-128 p/mg hair (P2.5-P97.5) [29].

### 2.5. Statistical Analysis

Differences between control vs. treated groups were analyzed using descriptive nonparametric statistics. Data were presented as median and range (minimal and maximal values). Mann–Whitney test was applied, and *p* < 0.05 was considered for significance. The GraphPad Prism 8.0 software was used for statistical analysis.

### 2.6. Ethics Aspects

This study was conducted following the Helsinki Declaration for medical studies in humans [30] and was approved by the Ethics Committee from the Faculty of Medicine of the University of Chile and the Guideline for good clinical practice [31]. Written informed consent was obtained from all volunteers.

## 3. Results

Hair cortisol was measured in samples obtained from 22 volunteers who met inclusion criteria. Volunteers were randomly divided into a control (*n* = 7) and a treated group (*n* = 15). The results found in the current study are shown in Table 1.

Initial sample collection was made two weeks after student's vacation period. The median of hair cortisol concentration in the control group was 1.8-fold higher after the treatment period, but in the treated group, the median was lower after the meditation activities. Meditation protocol was applied to subjects for three months. After that, a new hair sample was collected. Results show no significant statistical differences between control and treated groups neither in basal measures nor after meditation intervention (Figure 1(a)). However, cortisol values obtained before and after treatment in each subject show significant differences. The control group after the three months lasting this study shows higher cortisol levels. Individual differences in cortisol levels before and after the meditation course were calculated. The control group hair cortisol level median increased in 93 units pg/mg between basal and posttreatment. The meditation group showed a decrease in hair cortisol median of 30 pg/mg after meditation protocol application comparing to basal cortisol values (Figure 1(b)).

## 4. Discussion

The current study is aimed at evaluating the effects of a meditation intervention on hair cortisol concentrations as a chronic stress biomarker in an undergraduate student population of a medical faculty. Hair cortisol levels represent free cortisol percentage which diffuses from capillary blood to growing pilose follicles, incorporating into the hair, where it remains without degradation [29, 32]. The measurement of cortisol in hair is considered an excellent biomarker of chronic stress; its levels correlate positively with salivary cortisol, corroborated by many studies in the research about stressors affecting the population [33]. In our study, a hair sample was obtained in basal condition and after three months of occupational therapy intervention consisting in an active meditation protocol. In a previous study, Gonzalez et al. showed a hair cortisol concentration reference interval of 40-128 pg/mg hair (P.2.5-P.97.5) obtained in healthy individuals with low levels of stress.

The median obtained in the current study is considerably higher than the upper limit of the reference interval, yet it would be necessary to obtain a healthy reference range in the studied population to assess its actual significance. Results show that hair cortisol level was similar in both studied groups in basal conditions, but cortisol levels in the control group were higher after the study's intervention period. These findings suggest that during the course of the semester control group incremented their stress levels.

Meditation practice significantly prevents hair cortisol levels increase in the treated group, whose cortisol levels were similar before and after the studied period, indicating that meditation routines could help avoid academic-associated stress in undergraduate students. According to several authors, beneficial effects of meditation practice have been reported in different life scenarios [34–36]. Undergraduate education is one of the most relevant steps in people's development, but at the same time, it could be one of the most stressful ones. The control group showed increased stress. This may have been related to the exam period in which the whole group was involved and to a lesser extent to participating in a new activity (painting course) and having to acquire a new skill.

Our study does not have the tools to conclude that the control group's painting course induced a high degree of stress. However, both groups were subjected to academic evaluations related to their formal studies during the second sample was taken. Therefore, we suggest that the intervention of the meditation sessions prevented a higher degree of stress induced by the period of academic evaluations.

Different meditation-based strategies have been tested on people with stress-related illnesses showing promissory results in the same period of time [37, 38]. Medical care students are a relevant target to receive mental care through practices based on meditation or relaxation since there is evidence that occupational stress and burnout developed in healthcare personal. Mental and physical relaxation interventions could decrease 23% in stress levels compared to no intervention in healthcare workers [39, 40]. In this study, active meditation session effects were evaluated, and the result was beneficial. The incorporation of mind-body exercise, a mixture of bodily poses with meditation and breathing, has helpful goods on physical and mental health [41–43]. Specifically, mindfulness-based meditation practices are proved to be beneficial for appetite control [44], relax sensation [39], improving sleep disturbance [45, 46], and coping with daily situations [41]. Moreover, meditation has been incorporated in scholarly education reporting excellent results [15, 35]. Thus, it could be promissory to do that in undergraduate education, based on our results, at least to attenuate academic-associated stress.

The incorporation of meditation in students' daily routine through occupational therapy intervention reduces cortisol levels in hair, reflecting chronic stress. Here, we provide evidence on the benefits of integrating active meditation into the daily routine through an occupational therapy intervention, which could contribute to disease prevention and health promotion. It could be an exciting contribution into university context by developing strategies for adapting routine during the first year of university and improving stress-management.

Although the results do not indicate statistical significance, they prove that active meditation, through an occupational therapy program, is useful for coping with stressful situations. Although stress levels were not significantly reduced in the treated group, they were not increased in contrast to the control group. This shows the need for tools so that students can face stressful situations, which can contribute to maintaining their mental health and academic performance. On the other hand, Figure 1(b) shows the individually differences pre- and posttreatment. The reduction of cortisol level for each participant respects to their own basal value was significantly different, showing a beneficial result after meditation practicing. Meditation practicing requires personal training that could be influenced by the personal experience and learning of the technique, being necessary result interpretation individually and collectively.

## 5. Conclusions

Active meditation incorporation in the daily routine through occupational therapy intervention on a university student sample shows improvement on stress biomarkers such as hair cortisol concentration. This result raises questions about stress in students, mainly associated with academic environment and conditions.

Meditation activities are relevant to students' academic performance and could contribute to the prevention of diseases and the promotion of their health. This study gives evidence for incorporate active meditation in the curriculum of healthcare careers to improve the students' physiological, cognitive, and emotional states.

## 6. Limitations of the Study

Our study is limited to a restricted population group in terms of age and level of intellectual activity. It lacks a detailed study of environmental factors that could affect the students' stress levels. Among these factors, we can mention socioeconomic factors, the presence of diseases, or personal problems. Stress levels could be influenced by several factors not quantified in this study. On the other hand, we are aware that the meditation techniques used different protocols. However, they all had in common the body's movement and the control of consciousness. The results will allow us to design new studies focused on which meditation methods are more beneficial in reducing stress levels.

## Figures and Tables

**Figure 1:** Effect of active meditation practice on hair cortisol. (a) Hair cortisol was measured in basal conditions and after a 3-month meditation intervention (POST). (b) Individual hair cortisol differences between posttreatment and basal values. Data represent median ± range; Mann–Whitney test was performed; ^∗∗∗^*p* = 0.0003.

**Table 1:** Male and female distribution.

	Male	Female
Treatment group	1	14
Control group	2	5

**Table 2:** Distribution by year.

Study year	Control group	Treatment group
First year	8	4
Second year	1	1
Third year	3	1
Fourth year	3	1

**Table 3:** Hair cortisol levels in studied population. Data are presented as median and range between minimum and maximum, *n* = 22.

Group	Basal hair cortisol (pg/mg)	Postmeditation treatment hair cortisol (pg/mg)
Control	132 (83-273)	244 (94-749)
Treated	158 (63-481)	142 (40-423)

## Data Availability

The data used to support the findings of this study have not been made available because this information was not requested from the study participants, nor from the Ethics Committee; therefore, we are not in a position to share the data.
